The article "Artificial Intelligence-Based Semisupervised Self-Training Algorithm in Pathological Tissue Image Segmentation" was retracted in 2023. Reasons: unreliable results or conclusions; concerns about the data; concerns about the peer review; concerns about the citations.

# Artificial Intelligence-Based Semisupervised Self-Training Algorithm in Pathological Tissue Image Segmentation

**DOI:** 10.1155/2022/3500592

**Published:** 2022-06-13

**Authors:** Qun Li, Linlin Liu

**Affiliations:** ^1^School of Electronic Information Engineering, Ningbo Polytechnic, Ningbo 315800, China; ^2^School of Information and Engineering, China Jiliang University, Hangzhou 310000, Zhejiang, China

## Abstract

In the field of medical image processing, due to the differences in tissues, organs, and imaging methods, obtained medical images have significant differences. With the development of intelligence in medicine, an increasing number of computing optimization algorithms based on AI technology have also been applied to the field of medicine. Because the image segmentation algorithm based on the semisupervised self-training algorithm solves initialization class center large randomness problem in the traditional cluster-based image segmentation algorithm, this article aims to integrate the artificial intelligence semisupervised self-training algorithm into the pathological tissue image segmentation problem. An experimental group is designed to collect sample images and the algorithm proposed in this article is used to perform image segmentation to achieve a better visual experience and images. Although there is no general image segmentation theory, many scholars have been committed to applying new concepts and new methods to image segmentation in recent years and combining specific theoretical image segmentation methods has achieved good application results in image segmentation. For example, wavelet analysis, wavelet transform, neural networks, and genetic algorithms can effectively improve the segmentation effect. The results of the Seg cutting method designed in this article show that, in retinal blood vessel segmentation results on a database of healthy people, the sensitivity value is 0.941633, the false-positive rate is 0.952933, the specificity is 0.956787, and the accuracy rate is 0.96182, which are all higher than those in other methods. Image cutting methods such as FNN, CNN, and AWN have addressed the case tissue image cutting problem. Using the Seg cutting method designed in this article to segment the retinal blood vessels on a diabetes patient database, the sensitivity value is 0.8106, the false-positive rate is 0.0511, the specificity is 0.9712, the accuracy is 0.9421, and the false-positive rate is omitted. The false-positive rate is lower than AWN, and other indicators are higher than FNN, CNN, AWN, and other image cutting methods. The application of artificial intelligence-based semisupervised self-training algorithms in pathological tissue image segmentation is realized.

## 1. Introduction

Artificial intelligence refers to the use of artificial intelligence methods to perform mechanical intelligence, to simulate human intelligence on a machine, or to give humans machine intelligence. Since artificial intelligence occurs in machines, it can also be called mechanical intelligence. Because mechanical intelligence simulates human intelligence, it can also be called analog intelligence. At present, the term man-made consciousness is applied to “research on the best way to make human knowledge on machines.” In this sense, man-made consciousness is the investigation of how to construct savvy machines or canny frameworks to reproduce and broaden human knowledge. Man-made consciousness is the investigation of how to provide machines with the elements of tuning in, talking, perusing, composing, thinking, getting the hang of, adjusting to ecological changes, and tackling different issues. In rundown, man-made brainpower allows machines to perform undertakings that require human knowledge or more insight than people. Artificial intelligence algorithms are used in intelligent diagnosis and treatment, intelligent recognition of medical images, medical robots, and other medical aspects.

According to the dark-level quality of the image, at least one dark-level limit can be calculated using edge-based partitioning techniques, looking at the dark-level value of each pixel in the image with edges, and finally classifying the pixels into suitable categories for review. Each track on the disk is equally divided into several arc segments. These arc segments are the sectors of the disk. The reading and writing of the hard disk take the sector as the basic unit. In this way, the most basic advance of the strategy is to address the ideal dark limit as per a specific standard capacity. The region put together division strategy which is based on coordinate region search, and explicit calculations have local development, local detachment, and consolidation calculations. There are two basic types of region-based extraction strategies: one is that the local development gradually rises from an isolated pixel to form the necessary partitions; the other is that the expected partitioned regions are cut according to different perspectives around the world. By and by, division is typically a mix of these two essential structures, and it is great for the picture division of intricate scenes characterized by a few complex items or the division of a few normal articles. Generally, machine learning enables the machine to perform functions that cannot be achieved by direct programming; machine learning is the ability to use the collected data to train the corresponding model and then transmit the model information and make predictions. The two most important steps in machine learning are training and prediction, which can correspond to the induction and speculation process of human perception. Therefore, the machine learning process simulates the human learning process. The process of dealing with images is not a logical causal crisis but a related conclusion drawn through induction. Machine learning is deeply connected with pattern recognition, statistical learning, data mining, and other fields. Image segmentation refers to the image being divided into several areas according to grayscale, color, spatial texture, and other characteristics such as geometric texture or certain rules so that these characteristics in the same region show consistency or similarity and obvious differences exist between different regions. Image segmentation separates the parts of an image to facilitate further processing. The results of image segmentation are the basis for image understanding, such as image feature extraction and recognition.

The semisupervised self-training algorithm is the process of assisted clustering using sample data with labels or restricted information in the dataset, so the most important problem in the semisupervised self-training algorithm is how to effectively use the known labels or restriction information provided in the original data to guide the clustering process, which tends to obtain better results. It divides the data into different groups or classes and requires that the data in the same group have high similarity as much as possible, and the data between different groups have great differences. The semisupervised self-training image segmentation algorithm addresses the problem of the traditional clustering-based image segmentation, where the initialization class center has great randomness; it uses the idea of semisupervision to improve the clustering-based image segmentation algorithm and integrates limited artificial supervision information; that is, a few points on an image are selected to identify the corresponding region.

Semisupervised learning is a significant methodology in the example acknowledgment and AI field; a learning technique consolidates regulated learning and unaided learning. The examination subject of semisupervised learning is to utilize few named tests to mark an enormous number of unlabeled examples. With the persistent advancement of AI research and the rising fame of utilizing few marked examples to name an enormous number of unlabeled examples, semisupervised learning research has as of late turned into an exploration center.

As one of the medical image processing methods, medical image segmentation extracts the target object to the pixel point and uses image matching, artificial intelligence recognition, and modeling technology to reshape. Image input and image segmentation are interrelated. For example, when retina OCT is segmented, it is advantageous to accurately achieve a single-step ellipsoid zone (ellipsoid zone) to record the retina image, and the object can obtain a clear retina image without retrograde obstruction. According to the statistical results of journal and conference papers published in medical imaging in recent years, half of the medical imaging-related documents are pure image segmentation, one-quarter are image segmentation based on records, and one-quarter include segmentation and registration. This shows that medical image segmentation occupies an extremely important position in the image processing field. Guided learning is a method of learning according to prescribed procedures with systematic guidance. Guided learning can improve learning efficiency and help to achieve the two important teaching goals of effective learning: subject content and the continuous improvement of problem-solving skills. In many learning tasks, guided learning has a role for most students, but the necessity of this approach changes with the complexity and novelty of the knowledge or skills learned, as well as with individual experience and self-study ability. Guided learning has limitations. Some psychologists have suggested that it may be more appropriate to guide discovery learning with the advantages of both centralized and discovery learning in classroom learning.

Jeavons and Andrew proposed cotraining by a committee self-training learning framework. This method integrates three multiple classifiers for self-training learning, where the confidence is the average posterior probability of multiple classifiers. However, when selecting the maximum posterior probability, the repeated maximum posterior probability problem may arise [1]. In subsequent research, Davies proposed combining active learning and self-training methods to construct SVM classifiers. The SVM classifier is used to select samples with the category as the center, the rate of change in the label is 0, and active learning is used to select samples close to the decision limit. However, Davies' research did not solve the problem of using active learning to actively label self-training methods, which are difficult to determine [2]. From the work of Thrall et al., based on previous research, we substituted the algorithm into medical image analysis. Although they established a new active contour model by using the properties of spatial fuzzy clustering that successfully solved the problems of insufficient segmentation of microvessels and blood vessel intersections, it was more sensitive to initialization and could not be directly used for retinal blood vessel images with complex topological structures. Segmentation and the time overhead are large [3]. M Sipper et al. pointed out that artificial intelligence (AI) is a broad field dedicated to enabling machines to perform intelligent tasks; it has taken academia and industry by storm in an extremely short period of time [4]. JA Golden also stated that artificial intelligence (AI), the theory and development of computer systems capable of performing tasks that normally require human intelligence, permeates almost every aspect of modern life [5]. D. Hassabis and D. Kumaran et al., argued that the fields of neuroscience and artificial intelligence (AI) have a long and intertwined history, however, recently, communication and collaboration between the two fields has become less common. They believed that a better understanding of biological brains could play a crucial role in building intelligent machines [6]. H. Lu and Y. Li et al. stated that artificial intelligence (AI) is an important technology that supports daily social life and economic activities, and it has made great contributions to the sustainable development of the human economy and solved various social problems [7].

The innovations of this paper are as follows: (1) The algorithm combines active learning and self-training methods [8]. Active learning technology can intelligently use low-confidence samples to improve students' generalization ability. It uses experts to actively identify samples that the classifier cannot correctly classify, that is, samples with low confidence. (2) A new semisupervised data processing technology [9] is proposed. This data processing technology is based on semisupervised KNN as the basic classifier, which can use both labeled and unlabeled samples for data filtering [10]. (3) The designed algorithm can be successfully applied to the retina in actual ophthalmology clinics and initially solves the problem that there are few retinal segmentation algorithms that can be successfully applied in actual ophthalmology clinics.

## 2. Application Method of Artificial Intelligence-Based Semisupervised Self-Training Algorithm in Pathological Tissue Image Segmentation

### 2.1. Cascade Detection Method Based on a Classification Network

Because the cell morphology under normal conditions is very similar to the mitotic cell morphology, it is difficult to guarantee the accuracy and recall rate of a one-time test [11], so this paper studies the cascade test method [12]. The method used in this chapter first locates the candidate targets through the classification network and sliding window and roughly detects the candidate mitotic cells. In this step, we attempt to detect the cells that may be undergoing mitosis and then use the classification network to further screen out the mitotic cells and eliminate them. Similar to normal cells, the number of misdetected cells is reduced and accuracy is improved [13]. It is verified on the ICPR 2016 and 2018 datasets that this cascade detection method can achieve better detection results [14]. Mitosis is characterized by the presence of spindles and chromosomes in the process of cell division, so that the daughter chromosomes copied in S phase are evenly distributed to the daughter cells. This mode of division is widely seen in higher animals and plants (animals and higher plants). The mitosis of animal cells (lower plant cells) is different from that of higher plant cells.

Before using the cascade detection method, this article first refers to the deep neural network proposed by Cireşa et al., who won the ICPR 2016 competition, to build an 11-layer neural network, train the classifier, and use the classifier to detect most of the cells. Image segmentation is the technology and process of dividing the image into several specific and unique regions and putting forward the target of interest. It is a key step from image processing to image analysis. A large number of false-positive cells are also introduced [15]. It can be seen that training a classifier that only distinguishes mitotic cells from other regions cannot obtain better detection results. It must be based on the different characteristics of mitotic cells and normal cells and further screen out mitotic cells based on the detection results in Figure 1 [16]. Subsequently, this article utilizes the course discovery technique. To choose the grouping organization, the order precision of the 11-layer brain network in the approval set (marked information, not engaged with preparing, is utilized to check the arrangement exactness of the model) comes to 94%. The deep residual network selected in this paper (ResNet) through experiments showed that the accuracy rate on the verification set is as high as 98% [17]. The test results obtained are shown in Figure 1.

The cascade detection method based on the classification network uses ResNet to train two classifiers [18]. The first step is to automatically learn the characteristics of mitotic cells and the background, impurities, and normal cells through the CNN, train two rough classifiers [19], and then use sliding window scans to classify the image to detect candidate mitotic cells. The second step is to use the CNN to focus on learning the characteristics of mitotic cells and normal cells, training two accurate classifiers, and screening the candidate targets detected in the first step to reach the final test result [20].

### 2.2. Semisupervised Learning

Semisupervised learning is the major question in the example acknowledgment and AI field. A learning strategy joins administered learning and unaided learning. Semisupervised learning utilizes a lot of unlabeled information and all the while involves marked information for design acknowledgment. While semisupervised learning is utilized, it expects as couple of individuals as conceivable to accomplish the work and can likewise accomplish somewhat high precision. Therefore, semisupervised learning is receiving increasing attention. Clustering hypothesis means that examples in the same cluster are more likely to have the same tags.

Up to a suitable association in the unlabeled example dissemination in the preparation test set and the learning model classifier can be laid out, the unlabeled examples in the preparation test set can be completely used to help with further developing the learning execution of the classifier [21]. It is generally believed that this connection is achieved by using unlabeled samples in the training sample set to estimate the parameters in the generative model, but, in a more general case, it needs to be established based on certain assumptions in semisupervised learning; there is a connection between the unlabeled samples in the training sample set and the learning model [22]. At present, there are two common basic hypotheses in semisupervised learning: the clustering hypothesis and the manifold hypothesis [23]. False-positive results refer to the false interpretation of negative smears as positive, and false-negative results refer to the false interpretation of positive smears as negative. This belongs to the influence of technical factors.

Semisupervised learning uses a small number of labeled samples to label a large number of unlabeled samples. Currently, semisupervised learning methods are based on two hypotheses: hypothesis grouping and multiple hypotheses. The clustering hypothesis is based on the principle of globality, and the manifold hypothesis is based on the principle of locality.

The clustering hypothesis usually means that the sample examples in the same cluster are more likely to have the same sample category label [24]. According to the clustering hypothesis definition, the decision boundary of the sample category should be passed in an area with relatively sparse data; otherwise, the sample points in the dense area of the cluster may be divided into both sides of the category decision boundary. This is the mark for distinguishing the sample category [25]. Under the clustering hypothesis setting, the function of a large number of unlabeled samples in the training sample set is to divide the boundary between the dense and sparse regions of the data distribution in the sample space [26].

### 2.3. Semisupervised Self-Training Method and Algorithm Introduction

This paper uses semisupervised algorithm at the algorithm level. In the semisupervised method, we can train the classifier on a small amount of labeled data and then use the classifier to predict the unlabeled data. The efficiency of the algorithm is improved.

The naive Bayes classification model is based on Bayes' theorem. Let *X* be the observed sample data and let *Y* be the class label. The Bayesian formula is as follows:

(1) $$\begin{array}{c} P\left(Y|X\right)=\begin{array}{c} P\left(X|Y\right)P\left(Y\right)\\ P\left(X\right) \end{array}. \end{array}$$

Bayesian theorem is a theorem about the conditional probability (or marginal probability) of random events *a* and *B*, where *p* (*a* | *b*) is the possibility of *a* when *B* occurs, *P* (*Y* | *X*) is the posterior probability, *P* (*X* | *Y*) is the conditional probability, and *P* (*Y*) is the prior probability. To classify the unknown sample *x*_*t*_=(*x*_*t*1_, *x*_*t*2_,…, *x*_*tm*_), we must base it on the existing training set and calculate the prior probability, conditional probability, and total probability. The formula is as follows:

(2) $$\begin{array}{c} y_{t}=\underset{y_{i}\in Y}{\arg\max}\left(p\left(y_{i}|x_{t}\right)\right)=\left\{\begin{array}{c} p\left(x_{t}|y_{i}\right)p\left(y_{i}\right),\\ \sum_{j=1}^{\left|Y\right|}p\left(x_{t}|y_{i}\right)p\left(y_{j}\right). \end{array}\right. \end{array}$$

Naive Bayes assumes that the conditional probabilities are independent of each other. Then, the conditional probability is calculated as follows:

(3) Pxt|yi=∏j=1mpxtj|yi,Pxtj|yi=countx,tjyi,12πσxjie2σji2.

The prior probability is calculated as follows:

(4) $$\begin{array}{c} P\left(y_{i}\right)=\begin{array}{c} \left|y_{i}\right|\\ D \end{array}. \end{array}$$

The weighted KNN method design is carried out. Let *d*(*x*_*t*_, *x*_*i*_) (*i* = 1, 2,…, *k* + 1) be the distance between sample *x*_*t*_ and its *k* + 1 neighbors. WKNN uses the *k* + 1th neighbor to *x*_*t*_ to standardize the distances from the first *k* nearest neighbors to the *x*_*t*_ sample; then

(5) $$\begin{array}{c} D\left(x_{t},x_{i}\right)=\begin{array}{c} d\left(x_{t},x_{i}\right),\\ d\left(x_{t},x_{\left(k+1\right)}\right), \end{array}\left(i=1,\ldots ,k\right). \end{array}$$

SPSS (Statistical Product and Service Solutions), “Factual Products and Services Solutions” programming was initially called the “Sociologies Statistical Package” (Solutions Statistical Package for the Social Sciences); however, with the development of SPSS items and the profundity of administrations, SPSS formally changed its English title to “Measurable Product and Service Arrangements” in 2000, denoting a significant change in SPSS's essential heading. The overall names of SPSS for a progression of programming items and related administrations for measurable examination activities, information mining, prescient investigation, and choice help assignments are Windows and MacOSX. Then, we utilize the weighted part capacity to change the standard distance *x*_*t*_ into *x*_*i*_ and the comparative likelihood *p*(*x*_*i*_|*x*_*t*_) and acquire the following formula:

(6) $$\begin{array}{c} p\left(x_{i}|x_{t}\right)=\frac{1}{2\pi }\exp\left(-\frac{D\left(x_{t},x_{i}\right)}{2}\right). \end{array}$$

The back likelihood of *x*_*t*_ having a place with class *ω*_*r*_(*r*=1,2,…, *s*) is determined in view of the *k* closest neighbors of *x*_*t*_; then, at that point, we have the following formula:

(7) $$\begin{array}{c} P\left(y_{i}|x_{t}\right)=\frac{1}{\alpha }\sum_{i=1}^{k}\left(x_{i}|x_{t}\right)I\left(y==\omega_{r}\right),\\ I\left(A\right)=\left\{\begin{array}{cc} 1, & \text{true,}\\ 2, & \text{false,} \end{array}\right.\\ a=\sum_{i=1}^{N}P\left(x_{i}|x_{t}\right). \end{array}$$

The imported data obey a distribution composed of a mixture of *L* Gaussian distributions as in the following equation:

(8) $$\begin{array}{c} f\left(x|\theta \right)=\sum_{l=1}^{L}a_{l}f\left(x|\theta_{l}\right). \end{array}$$

The mutual information of introducing text feature *t* and category *c*_*j*_ is defined as follows:

(9) $$\begin{array}{c} \text{MI}\left(t,c_{i}\right)=\log\frac{p\left(t,c_{i}\right)}{p\left(t\right)p\left(c_{i}\right)}=\log\frac{p\left(t|c_{i}\right)}{p\left(t\right)}. \end{array}$$

The mutual information of feature *t* is obtained as follows:

(10) $$\begin{array}{c} \text{MI}\left(t\right)=\sum_{i=1}^{n}P\left(c_{i}\right)\log\frac{p\left(t|c_{i}\right)}{p\left(t\right)}. \end{array}$$

The algorithm is optimized to start the experiment. Picture division is a course of treating every pixel in the fragmented picture. Pixels for certain normal visual attributes have a similar mark. In picture division, a multidimensional vector can be used to represent a pixel, which looks more intuitive and convenient for data processing. Since picture division is a somewhat significant connection in picture handling, countless picture division calculations have been examined, yet the division impact of certain calculations is at times not great.

## 3. Application Experiment of Artificial Intelligence-Based Semisupervised Self-Training Algorithm in Pathological Tissue Image Segmentation

### 3.1. Image Segmentation and Related Concepts

Considering the problems of traditional image segmentation algorithms, the algorithm is combined with image segmentation, the traditional image segmentation algorithm is improved, and limited manual information is integrated; that is, the user selects a limited number of points on the image to identify the relationship between the corresponding regions. These identified points are regarded as the labeled information point set in semisupervised learning, and these few labeled information points are used to segment the remaining large number of unlabeled information points, thereby improving segmentation accuracy.

Picture division is the method and interaction of partitioning a picture into various explicit regions with remarkable properties and proposing objects of interest. It is a critical stage from picture handling to picture examination. The current picture division strategies are separated into the accompanying classes: limit-based division techniques, locale-based division techniques, edge-based division techniques, and division strategies in view of explicit hypotheses. According to a numerical perspective, picture division is the method involved with partitioning a computerized picture into disjoint regions. The course of picture division is additionally a stamping interaction; that is, the pixels having a place with a similar region are allocated a similar number. The purpose of image segmentation is to distinguish target pixels from background pixels. In the original image, the target is the distribution of branches and leaves, and the light-colored area is the background area. The segmentation algorithm needs to segment the dark branch area of the target. According to a numerical perspective, picture division is additionally a course of digitizing a picture and isolating it into commonly disjoint regions. The picture division process is the checking system, which consolidates similar traits. The regions are set apart with a similar list, as displayed in Figure 2.

After image segmentation, the target area is segmented, as shown in Figure 3.

Based on the above basic principles. This article uses fundus images in the HRF, STARE, and DRIVE databases as experimental data. Comparing the red, green, and blue channel images of the RGB fundus image, it is found that the green channel has more blood vessel information and higher contrast. Therefore, the green channel of fundus image is used as the experimental blood vessel segmentation. To make the segmentation more accurate, the GAC model is used to automatically obtain the “mask” of each retinal fundus image and stretch the limbs in the retinal fundus image. Then, the background of the retinal fundus image is calculated, the original image is removed, and the gray value is drawn. Then, the image is stretched to obtain a retinal blood vessel image with gray values inside a predetermined reach. In view of the investigation of Hessian rectangular anisotropy, Hessian matrix is often used in Newton method to solve optimization problems. Hessian matrix can be used to determine the extreme value of multivariate function. According to the eigenvalues and eigenvectors, this paper further develops the vascular response work, utilizes the vascular reaction capacity and edge to get an unpleasant blood fragment division picture, and uses this data to begin level change and build the past shape term, which conquers the accompanying issues: the defined level model is sensitive to initialization, while the regional energy adjustment term is sensitive to noise. In addition, the area, width, and height of the connecting sector are used to construct geometric operators to eliminate the smaller damage and artifacts of the connecting sector in the segmentation result of the defined horizontal model and to obtain the final segmented blood vessel image of the retina.

### 3.2. Training Set Design

The semisupervised self-training algorithm uses the sample data with labels or restricted information in the dataset to assist clustering. Therefore, the most important problem in the semisupervised self-training algorithm is how to effectively use the known labels provided in the original data or limit information, guide the clustering process, and use it to obtain better results. The image segmentation algorithm based on the semisupervised self-training algorithm addresses the problems of traditional cluster-based image segmentation algorithms. This problem is that the initialization class center has great randomness, and the semisupervised idea is used to improve the cluster-based image segmentation algorithm. Limited manual supervision information is integrated; that is, a limited number of points on the image are selected to identify the relationship between the corresponding regions, and these points are used as sample data with label information in the image segmentation algorithm based on a semisupervised self-training algorithm. These sample data are used to initialize the class center; that is, a small part of labeled data are used to assist a large amount of unlabeled data for clustering learning, thereby improving the algorithm performance.

The training set of the classification network includes images and corresponding category labels. The images in this article are RGB three-channel color images. The labels are 0 and 1, with 0 as a negative example and 1 as a positive example. In this method, to train two rough classifiers and two accurate classifiers, two different training sets need to be established, and an image block with a size of 101×101 is taken as the network input. An image block of this size can completely cover various forms of mitotic cells, ensuring that other cells are not covered.

The training set of the two rough classifiers contains two types of image blocks: mitosis and nonmitosis. The mitotic image block is used as a positive example. According to the ground truth label, the image block is intercepted with the coordinate point as the center, so that the mitotic cells fall in the center of the image. To make the positive example, the dataset is as diverse as possible, and the coordinate point of the mitotic cell edge is selected as the center so that the cells are distributed in various parts of the image block and are not limited to the center; the nonmitotic image block as a negative example excludes the remaining pixels after mitosis. The points are randomly sampled and intercepted, including background, impurities, and normal cells.

The training set of the two accurate classifiers contains two types of image blocks: mitotic cells and normal cells. Selecting positive examples is the same as that of the two rough classifiers. The difference is that the image blocks containing normal cells are selected for negative examples. Blue is used in the experiment. The ratio threshold method is used to screen out the cell area. The blue ratio threshold method is selected for the two following considerations. (1) The two precise classifiers extract the characteristics of mitotic cells and normal cells, and as many normal cells as possible are required as negative examples. The blue ratio threshold method algorithm is simple and it is easy to realize that, by adjusting the threshold, as many cell regions as possible can be selected to meet the requirements for making the training set. (2) Due to the uneven coloring of the dataset, using the same threshold has different effects on different pictures. The image blocks of each picture are extracted in a balanced manner, and different thresholds can be set for pictures with large color differences to ensure that the contributions of all pictures to the training set are relatively consistent.

### 3.3. Network Model Configuration

There are two important files for training a network model: the configuration file that defines the network structure and the solver file that sets the training parameters. This section explains the network configuration file adjusted for the training data.

The methods in this chapter are based on the ResNet 101 level. For the network data level (defining network input), this article converts the color image into the LMDB data format with higher reading performance as the network input. In the experiment, the average image value is subtracted for training and testing, which improves the speed and accuracy to a certain extent. The average of all training samples is calculated. Caffe provides the average data value calculated in the LMDB format and average file value in binary format.

The default input size of ResNet is 224 × 224, and the image size of the training set in this article is 101 × 101. Direct training causes the feature map dimension to be reduced to 1 before reaching the fully connected layer, and the subsequent convolution cannot be performed. The operation results in training failure. Zero padding can be performed on the input image to expand the size to 224 × 224. The size of the convolution step in one of the residual blocks is modified in this article so that the feature map has a different dimension after passing through this residual block. In this way, the network can adapt to the input of 101 × 101 size, which can be seen in the ResNet framework table listed above.

## 4. Application Analysis of Artificial Intelligence-Based Semisupervised Self-Training Algorithm in Pathological Tissue Image Segmentation

### 4.1. Data Description

The 2016 ICPR MITOSIS dataset comes from biopsy sections of the eyeballs of 5 volunteers from a Sydney hospital. After H&E staining, pathologists selected 10 high-magnification visual field images at 40x magnification from each patient's section. The slice area covered by the field of view map is 512 × 512, and the scanner digitizes with a resolution of 0.2456/pixel to obtain an RGB color picture with a resolution of 2084 × 2084. Considering the large image size, the step length of the sliding window is set to 5 in the experiment.

The entire dataset contains 50 pictures. Each picture provides a ground truth file in CSV format. The file gives the coordinates of each mitotic cell. The specific format is as follows. One line gives the coordinates of all pixels covered by a mitotic cell. In turn are the abscissa and ordinate of each pixel. Partial images of 20 slices from each patient are used as the training set, and the remaining photos are used as the test set. The training set contains 30 images, which contain a total of 221 mitotic cells, and the test set contains 14 images, which contain a total of 102 mitotic cells. The simulation of dynamic system is realized by calculating the state of continuous time steps within a specified time span. This calculation uses the information provided by the system model. The time step is the time interval at which the calculation occurs.

The result of a laboratory test or report is often expressed by (+) and (−). (+) and (−) here are not addition and subtraction signs in mathematical calculations but are used to indicate positive and negative results. Some people do not understand (+) and (−) as positive and negative. Sometimes, (+) can also indicate the severity of the development of a certain disease; that is, it represents the change in quantity.

Table 1 compares the detection results of the cascade detection method based on the classification network and other methods on the ICPR 2016 test set. The last line is the detection result of this article. Compared with other methods, the detection method in this paper increases the recall rate, that is, reduces the number of mitotic cells that are easily missed. The accuracy rate is not the highest; that is, there are more false-positive cells. Finally, the F-score is better than all methods except DRN.

Table 2 shows the detection and evaluation results of 5 sets of data in the test set. The first column contains 5 sets of data. The brackets indicate the number of images contained in this set of data. It can be seen in the table that there are large differences in the slice images between different patients, and the detection results obtained by the same method are also very different. The accuracy and recall rates of A06 and A09 are relatively high, and the detection effect is better. The accuracy of A08 and A16 is better, but the recall rate is very low, resulting in a low F-score. A13 contains only 2 mitotic cells, which are not detected, and the detection effect is the worst.

The monitoring effect of the cascade monitoring method based on the classification network is compared with other methods on the ICPR 2016 test set according to the F-score ranking from large to small, as shown in Table 3.

It can be seen in the table that the detection method in this paper has a certain improvement in both accuracy and recall rate, so the F-score is the highest.

Through the cell slice data statistics, the two cascade detection methods in this paper are compared in terms of detection accuracy and detection efficiency. The segmentation accuracy of SegNet is better than that of FCN. The detection accuracy of the two cascade detection methods on the ICPR 2016 dataset is shown in Figure 4.

Picture division is the essential issue of picture examination and example acknowledgment. It to a great extent decides the last investigation nature of the picture and the discriminant examination result. Picture division is a course of marking every pixel in a picture. This interaction gives pixels with similar mark a few normal visual attributes. The design is to streamline or change the picture portrayal, making the picture more clear and break down. As of late, countless picture division calculations have been investigated.

The second method improves the accuracy rate but loses the recall rate, and the final F-score is the same as that of the first method.

At long last, we think about the time utilization of the three techniques utilized on the ICPR 2016 dataset, which are the strategy proposed in this paper and the two exemplary division organizations: FCN and CNN. It very well may be found in the table that the course discovery technique in view of division and grouping abbreviates the identification time in the two stages, as displayed in Table 4.

It can be seen that the SegNet image segmentation method takes much less time in the first step compared to the previous two methods, which benefits from the integrated improvement of the algorithm in the first step.

### 4.2. Comparison of Image Enhancement Algorithms for Pathological Tissues

Comparing the edge expansion map of pathological tissue obtained by the algorithm in this paper with FCN, using the variance *S*^2^ of background image *I*_*Rvb*_ as an evaluation factor to measure background smoothness and noise level, and selecting pathological tissue images of diabetic patients and healthy people, the results are shown in Table 5.

It can be seen in Table 5 that, whether it is the bottom image of a healthy person or a diabetic patient, the blood vessel improvement image obtained by the algorithm in this document has a small change between the gray background values, which proves that the noise is in the document. The level of abnormal tissue images obtained is lower and more serious.

### 4.3. Quantitative Analysis of Segmentation Results of Different Algorithms

To further prove the retinal vessel segmentation performance of the algorithm in this article, the following large-scale retinal vessel segmentation experiments were carried out in the HRF, STARE, and DRIVE databases, and quantitative analysis was performed. By comparing the method in this article with algorithms that refer to various documents, we design parameters such as sensitivity, false-positive rate, specificity, accuracy, and F grade. A value of 0 means that there is no such indicator in the comparative literature.  Figure 5 shows the segmentation of retinal blood vessels in the normal individual database results.

Sensitivity refers to the ability of a device, equipment, or system to avoid performance degradation in the presence of electromagnetic disturbance; high sensitivity indicates low anti-interference ability. Sensitivity is a concept created by Joseph Nye and Keohane in the book “Rights and Interdependence” to analyze international politics. It refers to the size and speed of the dependence effect. It is used to describe how quickly a change in one part of the system will cause other parts to change.

Retinal blood vessels are an important part of the systemic microcirculation system, and changes in their morphological structure are closely related to the severity of cardiovascular diseases such as diabetes, hypertension, coronary arteriosclerosis, and cerebrovascular sclerosis. Diabetes is a global noncommunicable disease caused by retinopathy, which is the most common retinal vascular disease and is very prone to causing blindness. By extracting retinal vessels and the measurement and analysis of relevant parameters of features such as tube diameter and curvature, the prediction of diabetic retinopathy is possible to a large extent and, thus, to scientific implementation of preventive intervention and pharmacological treatment. Therefore, research on retinal image vascular segmentation technology is of great significance for medical clinical applications. The characteristics of retinal images are more complex and vary from person to person, and the automatic extraction of retinal blood vessels is extremely susceptible to external conditions and lesions. Therefore, improving the extraction accuracy of retinal blood vessels is an important research topic.

Figure 6 shows the results of retinal blood vessel segmentation in the database of diabetic patients.

Figure 6 shows that, in the retinal blood vessel segmentation results of the normal database, using the Seg cutting method designed in this article, the sensitivity value is 0.941633, the false-positive rate is 0.952933, the specificity is 0.956787, and the accuracy rate is 0.96182. They are all higher than the image cutting methods such as FNN, CNN, and AWN in the same period, and they solve the problem of image cutting of case tissues. As shown in Figure 6 and Table 6, using the Seg cutting method designed in this article, the retinal blood vessels can be segmented in the diabetic patient database, with a sensitivity value of 0.8106, a false-positive rate of 0.0511, a specificity of 0.9712, and an accuracy of 0.9421. The false-positive rate is lower than AWN, and other indicators are higher than FNN, CNN, AWN, and other image cutting methods. This proves that the Seg cutting method designed in this article has a good pathological image cutting effect in different groups of people, different pathological tissues, and different data types.

## 5. Conclusions

With the development of machine learning pattern recognition, especially the increasingly widespread clustering application in industrial production, how to effectively use the user's industry experience to guide the clustering tendency to improve clustering performance has become a trend in recent years. The user's industry experience is background knowledge. In the clustering process, identifying information is also called supervised information and prior information. The method of using supervised information to improve the performance of unsupervised clustering is called semisupervised clustering. It was shown that, applying the AI-based semisupervised self-training algorithm, the Seg image segmentation method to segment mid-pathological tissue images has a high retention rate compared to other types of image design methods, a shorter processing time, and more precise features in various parameters. This paper used the comparative analysis method and sample collection method, simplified the semisupervised self-training method's algorithm according to Bayes' theorem, and introduced the Seg image segmentation method based on the traditional Seg algorithm. The training set of the classification network included images and corresponding category labels. The images in this article were RGB three-channel color images. The labels were 0 and 1, with 0 as a negative example and 1 as a positive example. In this method, to train two rough classifiers and two accurate classifiers, two different training sets were established, and an image block with a size of 101 × 101 was taken as the network input. An image block of this size can completely cover various forms of mitotic cells, ensuring that other cells are not covered.

The results of the study showed that, in the retinal blood vessel segmentation results on a database of healthy people, using the Seg cutting method designed in this article, the sensitivity value was 0.941633, the false-positive rate was 0.952933, the specificity was 0.956787, and the accuracy rate was 0.96182, which are all higher than the other methods. Image cutting methods such as FNN, CNN, and AWN solved the case tissue image cutting problem. As shown in Figure 6, using the Seg cutting method designed in this article, in the retinal blood vessel segmentation results of the diabetic patient database, the sensitivity value was 0.8106, the false-positive rate was 0.0511, the specificity was 0.9712, and the accuracy was 0.9421. The false-positive rate was lower than AWN, and other indicators were higher than FNN, CNN, AWN, and other image cutting methods. Through experiments, it was shown that the image processing method designed in this article has a very good image cutting effect in different pathological groups, different pathological parts, and image databases of different formats. The shortcomings of this article are as follows: (1) The experimental data of this article were from ICPR 2016 competition data. In addition, the relevant competitions held by MICCAI in 2020 also provided experimental data. Due to the suspension of the evaluation results on the official website, this article was based on the 2020 MICCAI dataset. The results of the experiment have not been evaluated. Later, by opening the evaluation, the method of this article can continue to be verified, and these data can be combined to train a more generalized network model. (2) The algorithm designed in this paper is based on Bayes' theorem and does not seek reference or inspiration from other famous theorems. In follow-up research, we can refer to the experience of predecessors in many aspects and summarize the algorithm rules that are more suitable for the topic of this article. The next step can focus on the following aspects: image texture information, spatial information in the clustering process, manually selecting supervision data points, and assigning different weights to different data points. For color images, the algorithm's time complexity will be high; therefore, one of the goals is to optimize the algorithm process and reduce the time complexity.

## Figures and Tables

**Figure 1:** Deep neural network detection effect image.

**Figure 2:** Branch background image.

**Figure 3:** Background image of branches after image segmentation.

**Figure 4:** Comparison of the detection accuracy of two methods.

**Figure 5:** HRF_Healthy database retinal vessel segmentation results.

**Figure 6:** Diabetes database retinal blood vessel segmentation results.

**Table 1:** Comparison table of ICPR 2016 results of different methods.

	Precision	Recall	F-score
WARWICK	0.451	0.573	0.514
UTRECHT	0.511	0.681	0.582
NEC	0.741	0.591	0.654
IPAL	0.691	0.741	0.718
DNN (Deep Neural Networks)	0.881	0.700	0.783
DRN (Distributed Routing Network)	0.789	0.802	0.791
**CNN (Cable News Network) + SW (ours)**	**0.734**	**0.854**	**0.789**

**Table 2:** Test set evaluation results.

Number	TP	FP	FN	Precision	Recall	F-score
Slide A06	38	5	26	0.601	0.883	0.718
Slide A08	31	33	24	0.564	0.483	0.520
Slide A09	41	21	13	0.766	0.651	0.704
Slide A13	0	4	2	0	0	—
Slide A16	29	44	3	0.904	0.396	0.553

**Table 3:** ICPR 2016 results comparison table of different methods.

Method	Precision	Recall	F-score
STRASBOURG	—	—	0.024
YILDIZ	—	—	0.167
MINES-CURIE	—	—	0.235
CUHK	—	—	0.356
RCasNN	0.361	0.423	0.389
CasNN	0.460	0.507	0.483
**CNN** **+** **SW (ours)**	**0.561**	**0.674**	**0.613**

**Table 4:** Comparison of the detection efficiency of the two methods.

Method	The first step is the detection time required per photo	The second step is the detection time required per photo (s)
CNN + SW	20 mins	4.2891
FCN + CNN	165.2181 s	1.7579
SegNet + CNN	1.10193 s	1.6127

**Table 5:** Comparison between the algorithm in this paper and the variance in the blood vessel enhancement image obtained by FCN (fully convolutional networks).

HRF_healthy	a	b	c	d	e
SegNet + CNN	71.9248	95.0557	81.6188	57.3821	59.1564
FCN	106.3369	112.8018	157.8544	91.5548	101.3254
HRF_healthy	A	B	C	D	E
SegNet + CNN	73.4818	175.9354	70.3381	82.4703	193.1479
FCN	177.9209	254.7669	77.3720	168.5366	191.3804

**Table 6:** Comparison of the effectiveness of the Seg cutting method between healthy and diabetic patients.

Seg cutting method	Sensitivity	False-positive	Specificity	Accuracy
Normal person database	0.941633	0.952933	0.956787	0.96182
Diabetes database	0.8106	0.0511	0.9712	0.9421

## Data Availability

No data were used to support this study.
